# MAGAN: Mask Attention Generative Adversarial Network for Liver Tumor CT Image Synthesis

**DOI:** 10.1155/2021/6675259

**Published:** 2021-01-30

**Authors:** Yang Liu, Lu Meng, Jianping Zhong

**Affiliations:** ^1^Shenyang Institute of Automation, Chinese Academy of Sciences, Shenyang 110000, China; ^2^College of Information Science and Engineering, Northeastern University, Shenyang 110000, China

## Abstract

For deep learning, the size of the dataset greatly affects the final training effect. However, in the field of computer-aided diagnosis, medical image datasets are often limited and even scarce. We aim to synthesize medical images and enlarge the size of the medical image dataset. In the present study, we synthesized the liver CT images with a tumor based on the mask attention generative adversarial network (MAGAN). We masked the pixels of the liver tumor in the image as the attention map. And both the original image and attention map were loaded into the generator network to obtain the synthesized images. Then, the original images, the attention map, and the synthesized images were all loaded into the discriminator network to determine if the synthesized images were real or fake. Finally, we can use the generator network to synthesize liver CT images with a tumor. The experiments showed that our method outperformed the other state-of-the-art methods and can achieve a mean peak signal-to-noise ratio (PSNR) of 64.72 dB. All these results indicated that our method can synthesize liver CT images with a tumor and build a large medical image dataset, which may facilitate the progress of medical image analysis and computer-aided diagnosis. An earlier version of our study has been presented as a preprint in the following link: https://www.researchsquare.com/article/rs-41685/v1.

## 1. Introduction

Medical image analysis and processing is the core of computer-aided diagnosis, which has been greatly prompted by deep learning. And the training of deep learning can be extensively influenced by the size of the dataset; that is, the more datasets can be obtained, the better the performance the trained deep learning model can achieve. However, in the field of computer-aided diagnosis, the medical image is very limited and even scarce, due to the privacy of patients, the expense of medical image acquisition, and so on. Therefore, synthesized medical images can be seen as the only feasible way to solve this problem, and generative adversarial networks (GAN) [1, 2] provide us a powerful tool to realize it.

GAN was firstly proposed by Goodfellow and colleagues in 2014 and was widely used in various fields, such as image processing, natural language processing, and even medical image synthesis [3]. For skin lesion images, Baur and colleagues synthesized the images of skin lesions with GAN [4], which enlarged the skin image dataset and improved the performance of lesion segmentation. For liver CT images, GAN was mainly used for expanding the dataset of the liver lesion [5] or image denoising [6], but the focus of GAN was only on the liver lesion, not on the whole liver CT images. For brain images [7], there are many image modules, such as CT images, magnetic resonance (MR) images, and positron emission tomography (PET), and different modules have different image acquisition methods and different influences on human brains. Dong Nie and colleagues used GAN to synthesize 7T images from 3T MR images [8] because 7T magnetic resonance (MR) images were very rare due to the expensive image acquisition costs and the side effects of high magnetic field strength. Moreover, some studies proposed to train a GAN to generate CT images from MR images to avoid the radiation from the CT image acquisition [9, 10]. For retinal images, the image resolutions were generally smaller than 100 × 100, and the image contents were only limited to single color background and vessels. Based on the characteristics, some studies [11] used GAN to synthesize the whole retinal image to enlarge the retinal image dataset, but the method cannot be generalized to other medical image modules with bigger image resolution and more organs, such as liver CT image or brain MR image.

Above all, all these medical image synthesis methods can be categorized into three types: (1) transformation of different modules, such as from CT images to MR images, (2) transformation between the different parameter of image acquisition, such as from 3T MR images to 7T MR images, and (3) image synthesis of the small resolution, such as skin and retinal images. Although there were many existing methods, medical image synthesis is far from clinical applications, since there are still some shortcoming.

### 1.1. Image Resolution

Many current medical image synthesis methods can only synthesize images with low resolution, which were lower than 128 × 128. However, most of the medical images in the clinical application were high image resolution, such as 512 × 512 CT images and 512 × 512 MR images.

### 1.2. Lesions or Tumors

The current existing medical image synthesis methods cannot synthesize images with abnormalities, such as liver lesions and liver tumors. As we know, the size and variety of the training dataset are essential to the performance of deep learning methods. During the training of medical images' classification and analysis, it was essential to have both normal images and abnormal images to create an effective data set, but the medical images with abnormalities were relatively rare due to the hospital policy, patients' privacy, and so on. Therefore, synthesizing medical images with abnormalities can enlarge the dataset of deep learning methods and upgrade the performance.

To solve the shortcomings, we proposed a novel image synthesis model for normal liver CT images and liver CT images with tumors based on mask attention generative adversarial network (MAGAN). Using this model, we can build a liver CT image dataset consisting of thousands of synthesized 512 × 512 slices; furthermore, it also can facilitate the progress of computer-aided diagnosis and the training of deep learning models.

The main contributions of our work are as follows: (1) we combined GAN with attention mechanism and proposed a novel MAGAN model and (2) we proposed an effective method of enlarging the existing medical image dataset.

## 2. Materials and Methods

In the present study, we synthesized liver CT images with tumors based on the mask attention generative adversarial network (MAGAN) model [12], whose framework is shown in Figure 1. Firstly, all the pixels of liver tumors in the original image were labeled by the white color and used as the attention map. According to the attention mechanism, liver tumors were the highlighted relevant features of the CT images, and the attention map was also the key part of the success of the proposed algorithm. In the procedure of image synthesis, the liver tumor was the saliency map in the whole liver CT image, which meant that all the pixels of the liver tumors were masked by the attention map. The original image and the attention map were paired together and called “pairing A.” Then, the original image and the attention map were loaded into the generator network to obtain a synthesized image, and the attention map and the synthesized image were paired together and called “pairing B.” Next, pairing A and pairing B were both loaded into the discriminator network to determine if the synthesized image was real or fake. The generator network and the discriminator network were trained with adversarial learning so that both of them can become more and more powerful. After training, the generator network can fill the pixels of the attention map with similar gray values, texture, and shape of liver tumors, to synthesize liver CT images with tumors. More details of our model can be obtained from Sections 2.1∼2.3.

### 2.1. Attention Model

All liver CT images used in our method were from a public liver CT dataset, Liver Tumor Segmentation (LiTS) [13, 14], which was from the MICCAI 2017 competition. In the LiTS dataset, the pixel distance was from 0.55 mm to 1.0 mm, the slice spacing was from 0.45 mm to 6.0 mm, and the image resolution was 512 × 512. LiTS consisted of 131 enhanced CT image sequences, and all the tumors in the liver CT images were manually labeled by radiologists. We aimed to synthesize liver CT images with tumors, and the synthesized materials were from two aspects, liver CT images from healthy controls and liver tumor CT images from patients. Moreover, the liver tumor was the most salient region for clinicians and was also the most difficult part of the whole synthesis procedure. Therefore, according to the tumor labels from the LiTS dataset, the image values of all the corresponding pixels in the tumors were changed to 4096, which meant “white color,” and represented as an attention map in our model. Based on the attention mechanism, the original image and the attention map were transformed into feature maps *A* and *B* by using 1 × 1 convolution, respectively, and then all these feature maps were concatenated by using matrix multiplication, shown in Figure 2:

(1) $$\begin{array}{c} S_{i,j}=A_{i}^{T}B_{j}. \end{array}$$

Then, we performed softmax on the concatenated feature maps *S*_*i,j*_ to calculate the distribution of attention *D*_*i,j*_ on the *i*th position of the *j*th synthetic region:

(2) $$\begin{array}{c} D_{i,j}=\frac{\exp\left(s_{i,j}\right)}{\sum_{i=1}^{N}\exp\left(s_{i,j}\right)}. \end{array}$$

Therefore, the liver tumor mask images were used as attention maps to efficiently find the liver tumors' internal and external characteristics of the images.

### 2.2. Generator Network

The structure of our generator network is shown in Figure 3, which consisted of two contracting paths and an expansive path, showing the U-shape architecture [15]. The input of these two contracting paths was the original image and attention map, respectively; both of them consisted of nine blocks, and each block was composed of the ReLu layer, convolutional layer, and batch normalization (BN) layer.

In the contracting path, the image resolution was reduced but the feature information was increased. To overcome the drawback of a regular convolution operator, whose receptive field was small, we used a dilated convolution operator [16] in the first four layers of the contracting path, so that we can capture image features from a larger scale. And we used a regular convolution operator in the other five layers of the contracting path because the sizes of the images were already smaller than 32 × 32, which cannot support a dilated convolution operator. The feature maps from both of the two contracting paths were firstly loaded as input to the attention model, whose framework is shown in Figure 2, and then the distribution of attention value was transferred via residual connections. In the expansive path, the spatial information and the feature information were combined through a sequence of upconvolutions layer, BN layer, ReLu layer, and residual connections with high-resolution features from the attention model. Residual connections played important roles in MAGAN, which were used to bypass the nonlinear transformation, accelerate the training speed, and upgrade the performance of our model in the training of the deep CNN.

512 × 512 original image and attention map were loaded as inputs into the generator network, and the image resolution was reduced by half while passing each block in the contracting path. After nine blocks in the contracting path, the input images became 1 × 1 with 1024 feature maps. Then, these feature maps were upconvolved in the expansive path, and the size of the image increased one time while passing each block in the expansive path. After nine blocks in the expansive path, the image was restored as a 512 × 512 resolution image. In the generator network, the whitened regions in the liver CT images can be transformed into tumor regions. The loss function of our generator network is shown as the following formula:

(3) $$\begin{array}{c} L_{\text{adv}}\left(G\right)={Ε}_{v,r∼p_{\text{data}}\left(v,r\right)}\left[{\left\|r-G\left(v\right)\right\|}_{1}\right], \end{array}$$

where *r* denotes the real image, *v* denotes the concatenated image, and *G*(*v*) denotes the synthesized image calculated by the generator network.

### 2.3. Discriminator Network

The structure of our discriminator network is shown in Figure 4, which consisted of six blocks, and each block was composed of a convolutional layer, ReLu layer, BN layer, or sigmoid layer.

The inputs of the discriminator network were two pairings, which were pairing A (original image, attention map) and pairing B (synthesized image, attention map). Inspired by PatchGAN [12], all the 512 × 512 resolution images were divided into 900 patches, whose size was 142 × 142. After going through six blocks of the discriminator network, the sizes of output probabilities maps were 30 × 30, which indicated each pixel in the output probabilities maps corresponded to one patch of the input images. The mean value of all the pixels in the probabilities maps can be recognized as the result of the discriminator network.

The loss function of our discriminator network is shown as the following formula:

(4) $$\begin{array}{c} L_{\text{adv}}\left(D\right)=E_{v,r∼p_{\text{data}}\left(v,r\right)}\left[\log\;D{\left(v,r\right)}_{\text{real}}\right]+E_{v∼p_{\text{data}}\left(v\right)}\left[\log\left(1-D{\left(v,G\left(v,r\right)\right)}_{\text{fake}}\right)\right], \end{array}$$

where *r* denotes the real image, *v* denotes the attention map, *G*(*v*, *r*) denotes the synthesized image calculated by the generator network, and *D*(*v*, *r*) denotes the discrimination probability calculated by the discriminator network.

The total loss function of our GAN is shown as the following formula:

(5) $$\begin{array}{c} L=\arg\underset{G}{\min}\underset{D}{\max}\lambda_{1}L_{\text{adv}}\left(G\right)+\lambda_{2}L_{\text{adv}}\left(D\right), \end{array}$$

where *λ*_1_ and *λ*_2_ are coefficients.

## 3. Results

In our experiments, we used LiTS as our image dataset of liver CT images with tumors, which consisted of only 131 sequences. The size of LiTS was not big enough for the training of deep learning algorithms, such as liver tumor segmentation or classification. To enlarge the LiTS, we chose 4555 2D slices with tumors from 131 sequences of liver CT images. Then, all the images were normalized by using the following formula:

(6) $$\begin{array}{c} {\text{value}}_{\text{normalized}}=\frac{{\text{value}}_{\text{original}}-\text{mean}}{\text{std}}, \end{array}$$

where value_original_ and value_normalized_ represent the original and normalized image pixels value, respectively. Mean indicate the mean value of image pixels, and std indicate the standard deviation of image pixels. Moreover, we specially cut the tumor regions from the liver CT images and built a liver tumor dataset; then, we augmented the tumor dataset by flipping, rotating, and scaling the original tumor region so that we can create a liver tumor dataset of 50000 slices from the original 4555 slices, which were used as the mask attention map in our method.

The hardware and software configuration of our experiments are shown in Table 1. The quantitative evaluation metric used in our experiments was the peak signal to noise ratio (PSNR). There were four sections in our experiments, including training of our model, quantitative comparison between our method and other state-of-the-art methods, Turing test for the synthesized images by radiologists, and the evaluation of the synthetic dataset for the medical image segmentation.

### 3.1. Training of Our Model

The configurations of hyperparameters in our model during the training are shown in Table 2. The proposed MAGAN network was implemented by Python 2.7 and TensorFlow 1.1 and trained on an NVIDIA GeForce GTX 1080 GPU using Adam optimizer with a learning rate of 0.0002. It costs about ten hours for the whole procedure of the training.

As shown in Figures 5(a)–5(d), we can find that, as the number of iterations increased, the performance of the synthesized CT liver images became better and better. After the first iteration of training (in Figure 5(a)), the performance of the synthesized image from the generator network was terrible; for example, most pixels were black and the contour was blurring, intense chessboard effect. All these bad performances indicated that the training had just started, and more iterations were needed. After ten iterations (in Figure 5(b)), the whole image was more clear, the contour was more vivid, but the chessboard effect still existed. After one hundred iterations (in Figure 5(c)), the performance of the synthesized image was much better and closer to the real image, more details can be visualized, human organs were vivid, the chessboard effect was weaker but still existed, and whitened regions were not filled with tumor texture. After one thousand iterations (in Figure 5(d)), the chessboard effect disappeared, all details of liver CT were restored, and it was hard to tell the differences between synthesized image and real image.

The loss function of the generator network, discriminator network, and total network during the training is shown in Figures 6–8, respectively, and we can conclude that the loss functions decreased as the number of iterations increased and became steady after about 10000 iterations, which indicated that our model performed well during the training.

Results of the synthesized image are shown in Figure 9: three liver tumor images with tumor masks were in the first row, which was used as inputs of our model, and we can obtain the synthesized images in the second row. We compared the synthesized images and the real images and calculated the differences between them. The color image of the differences is shown in the fourth row. All these results showed that our method can synthesize liver CT images with tumors, and the synthesized images were almost identical to the real images.

To test the impact of the dilated convolution operators in the MAGAN, we replaced the dilated convolution operators with the regular convolution operators in the contracting path of the generator network and quantitatively compared the PSNR of these two GAN networks. And we found that the network with regular convolution operators can provide a PSNR of 59.66, while the MAGAN with dilated convolution operators can provide a PSNR of 64.72, which indicated the effectiveness of the dilated convolution operators in our network.

To test the impact of the residual connections in the MAGAN, we removed the residual connections and quantitatively compared the PSNR of these two GAN networks. And we found that the network without residual connections can provide a PSNR of 55.23, while the MAGAN with residual connections can provide a PSNR of 64.72, which indicated the effectiveness of the residual connections in our network. The running time of the proposed method was 0.087 seconds per frame.

Besides, we can also manually or automatically “add” tumor regions on the healthy liver CT images using our liver tumor dataset of 50000 slices, to create a diseased liver CT image, shown in Figure 10. The healthy liver CT images were in the first row. In the second row, manually change the pixel values of two regions to white color, which meant that these two regions were the selected tumor regions. Using our method, the results of the synthesized images are shown in the third row. All these results showed that our method can intelligently create liver CT images with tumors based on the healthy liver CT images, and the synthesized diseased images were almost identical to the real ones.

### 3.2. Quantitative Comparison

In this section, we quantitatively compared our method with other seven state-of-the-art medical synthesis methods using the same dataset as ours: (1) atlas-based method [17]; (2) sparse representation (SR) based method; (3) structured random forest with ACM (SRF+) [18]; (4) manipulable object synthesis (MOS) [19]; (5) deep convolutional adversarial networks (DCAN) method [8]; (6) multiconditional GAN(MC-GAN) [20]; and (7) mask embedding in conditional GAN (ME-cGAN) [21]. The first four methods were implemented by our group, and the source codes of DCAN, MOS, and ME-cGAN were downloaded from GitHub (http://www.github.com/ginobilinie/medSynthesis, http://www.github.com/HYOJINPARK/MC_GAN, and http://www.github.com/johnryh/Face_Embedding_GAN). The results of the quantitative comparison are shown in Table 3, which indicate that our method outperformed the other seven approaches and benefited from attention mechanism, dilated convolution operator, and residual connections.

### 3.3. Turing Test

To further verify the effectiveness of our method, we did the Turing test. Two experienced radiologists from Shengjing Hospital of China Medical University were asked to classify one hundred liver CT images into two types: real image or synthesized image. The radiologists were not aware of the answer to each image before the Turing test. The one hundred liver CT images consisted of fifty real CT images and fifty synthesized images. The results of the Turing test are shown in Table 4: radiologist number 1 made correct judgments for 74% real image slices and 64% synthesized image slices and radiologist number 2 made correct judgments for 84% real image slices and 12% synthesized image slices. The radiologists made correct judgments for most of the real images and may be psychologically influenced by the existence of a synthesized image, so they made some errors about the real images. Furthermore, the radiologists made difficult judgments for the synthesized images and cannot tell the obvious differences between the real images and the synthesized images. And according to radiologist #1, his most reliable evidence of telling the difference was the color of the tumor region was a little darker than the real ones, which was also the improvement we needed to do in the future. All these results of the Turing test indicated that our method can synthesize liver CT images with a tumor, which were almost identical to the real ones.

### 3.4. Evaluation of Synthetic Dataset for Medical Image Segmentation

To evaluate the effectiveness of the synthetic dataset in the training of deep learning models, we used a fully connected network (FCN) [15] to perform the tumor segmentation task in the liver CT images and trained the FCN model using the LiTS dataset (images from 131 subjects) and the new dataset obtained by our method (images from 131 real subjects and 865 synthetic subjects). And we used the Dice Index to quantitatively evaluate the performance of the segmentation results from the two trained FCN models. The FCN model trained by the LiTS dataset can provide a Dice value of 0.611 for the tumor segmentation, and the FCN model trained by a new dataset can provide a Dice value of 0.658 for the tumor segmentation. The result indicated that the synthesized liver CT images obtained by the proposed method can effectively enlarge the original dataset, and as the number of images in the dataset increased, the performance of the training of the deep learning model can become better, which resulted in the higher Dice value for the liver tumor segmentation.

## 4. Discussion

In the present study, we combined the attention mechanism and GAN model and proposed a novel CT image synthesis algorithm, which was MAGAN. As far as we know, the existing medical image synthesis methods mainly focused on the transformation of different modules or transformation between the different parameter of image acquisition, and our study was the first research of synthesizing the liver CT images with tumors in high resolution and enlarging the size of the medical image dataset.

Suppose that we had a dataset of chest CT images with lung nodules, whose size was one hundred. While we used this dataset for the training of deep learning, we may find that the trained model was not good enough due to the small size of the dataset. Under these circumstances, the proposed MAGAN can be used to synthesize thousands of chest CT images with lung nodules based on the original one hundred images. This kind of similar requirements from clinical researches and deep learning studies is very common. And the proposed method can meet the requirements.

From the quantitative comparison between the proposed method and the other seven state-of-the-art medical image synthesized methods, we can conclude that the proposed method outperforms the others, and the main reasons were the attention map, which mainly focused on the regions of interest in the medical images, such as liver tumors or lung nodules.

During the Turing test, two experienced radiologists cannot clearly distinguish the synthesized liver CT images and the real liver CT images. We used the judgments of experts as the golden standard, and we may conclude that the synthesized liver CT images with tumors can be used as the real ones, and the size of the training dataset of medical images can be enlarged from one hundred to thousands. The bigger the medical image dataset is, the better the training performance can be.

## 5. Conclusions

In the present study, we proposed a method of synthesizing liver CT images with tumors based on mask attention generative adversarial networks. The experimental results showed that our method outperformed the other seven widely used approaches and can achieve 64.72 db mean PSNR, and the Turing test indicated that even the experienced radiologists cannot tell the differences between the synthesized images from our method and the real ones. All these results meant that, using our method, we can build a huge medical image dataset to facilitate the diagnosis of computer-aided diagnosis and the training of deep learning.

## Figures and Tables

**Figure 1:** The framework of our model: ⊗ represents matrix multiplication.

**Figure 2:** The framework of the attention model.

**Figure 3:** The framework of our generator network.

**Figure 4:** The framework of our discriminator network.

**Figure 5:** Synthesized image during the training of the proposed model: (a) after one iteration of training, (b) after ten iterations of training, (c) after one hundred iterations of training, (d) after one thousand iterations of training.

**Figure 6:** The loss function of the generator network during the training.

**Figure 7:** The loss function of the discriminator network during the training.

**Figure 8:** The loss function of the total network during the training.

**Figure 9:** Results of the synthesized images and the comparison between the synthesized images and real images. The pixel values of the fourth rows are weak and low because the differences between the real images and synthesized images were very small.

**Figure 10:** Adding tumor regions on the healthy liver CT images and synthesizing diseased liver CT images using our method.

**Table 1:** Hardware and software configuration of our experiments.

Item	Configuration
Operating system	Ubuntu 16.04
GPU	NVIDIA GeForce GTX 1080
CPU	Intel Core i5-7500 @3.4 GHz
Software toolkit	Python 2.7; TensorFlow 1.1; MATLAB 2016b
Disk	500 GB
GPU memory	8 GB
System memory	16 GB

**Table 2:** Hyperparameters of our model.

Parameter	Value
Initial learning rate	0.0002
Adam momentum	0.5
*λ*_1_ in formula (5)	100
*λ*_2_ in formula (5)	1
Exponential decay	0.99
Batch_size	1
Epoch	10
Dropout	0.5
Frequency of saving loss value	100
Frequency of saving model	500

**Table 3:** The quantitative comparison between our method and seven other approaches.

	Method							
	Atlas [17]	SR	SRF+ [18]	MOS [19]	DCAN [8]	MC-GAN [20]	ME-cGAN [21]	Our method
Mean PSNR(dB)	45.15	49.77	55.30	60.11	58.26	59.29	61.35	64.72

**Table 4:** The Turing test of our method.

	Real image (50 slices)		Synthesized image (50 slices)	
	Be judged as real images	Be judged as synthesized images	Be judged as real images	Be judged as synthesized images
Radiologist number 1	37	13	18	32
Radiologist number 2	42	8	44	6

## Data Availability

Liver CT images used in our method were from a public liver CT dataset, which is Liver Tumor Segmentation (LiTS), and the data can be obtained from https://academictorrents.com/details/27772adef6f563a1ecc0ae19a528b956e6c803ce.
